The article "Comprehensive Evaluation of the Tendency of Vertical Collusion in Construction Bidding Based on Deep Neural Network" was published in 2022. Journal: Comput Intell Neurosci.

# Comprehensive Evaluation of the Tendency of Vertical Collusion in Construction Bidding Based on Deep Neural Network

**DOI:** 10.1155/2022/2897672

**Published:** 2022-07-13

**Authors:** Wenxi Zhu, Kaizhi Cheng, Yabin Guo, Yun Chen

**Affiliations:** ^1^School of Traffic and Transportation Engineering, Changsha University of Science and Technology, Changsha 410114, China; ^2^Key Laboratory of Highway Engineering (Changsha University of Science & Technology), Ministry of Education, Changsha, China; ^3^Yunji Smart Engineering Co., Ltd., Shenzhen 518000, China

## Abstract

To effectively diagnose and monitor the vertical collusion in construction project bidding, this paper developed a comprehensive evaluation model with deep neural network and transfer learning. By this model, the collusion characteristics of bidders, tenderers, and bid evaluation experts were mined from limited data set hidden and collusion tendency was evaluated. Firstly, 18 evaluation indicators were established from literature review, court file summarization, typical case analysis, and expert consultation. Then, a comprehensive evaluation model was developed with the deep neural network and transfer learning. Finally, the model was trained and tested with the collected data set. The test results showed that the developed model achieved 87.3% identification accuracy in collusion tendency evaluation of different subjects.

## 1. Introduction

There are many problems in the process of project construction, especially the collusion phenomenon in the bidding stage [1, 2]. In addition, the collusion in bidding has become more and more prominent due to factors such as information asymmetry, inadequate supervision, imperfect system, and unscientific management [3], and the concealment and non-detectability of the bidding collusion in construction projects are gradually increasing [4].

For the problem of vertical collusion in bidding for construction projects, a lot of research has been conducted by scholars, mainly including: in terms of the motivation of collusion behavior, Aoyagi [5] deduced the equilibrium conditions of collusion between bidders and tenderers and analyzed the distribution of benefits after collusion; Zarkada-Fraser and Skitmore [6] studied the factors influencing bidder collusion based on their psychology, attitude, and behavior when colluding; Pesendorfer [7] stated that the two main ways of tenderer-bidder collusion were compensation and subcontracting; Lugovskyy et al. [8] stated that cooperation experience, reputation, and initiative were the main factors that lead to collusion between regulators and bidders; Dotoli et al. [9] showed that inadequate government oversight of bidding collusion and low penalty costs led to invalid oversight and occurred collusion; Friedman [10] found that the high rate of return (financial interest) was the underlying motive for collusion by analyzing the causes of collusion. Scholars also found that the psychology of the participants had some influence on collusive bidding [11]; cost asymmetry and unreasonable offers were the “triggers“ for collusion [12, 13]. In terms of collusion prevention, Zhang [14] analyzed the possibility of collusion based on the project properties, market environment, collusion costs, and collusion benefits, and also constructed a three-party game model, which showed that reducing regulatory costs, improving regulatory tools, increasing penalties, and benefits for participants can strongly curb collusion; Cavill and Cavill [15] pointed out that strengthening the accountability of the stakeholders involved in bidding, improving their respective responsibilities, and efficiently fulfilling their obligations have important effects on preventing the collusion; Rahman et al. [16] emphasized the importance of maintaining information symmetry, guaranteeing information security, and preserving data privacy in the process of against collusion, and proposed the signing of privacy bid agreement as a governance measure; Boone and Mulherin [17] and Ishiguro [18] indicated that the fundamental way to eliminate the occurrence of collusion in bidding was to establish a bidding supervisory body and gave full play to the regulatory role of the acting government, and handled timely for supervision efficiency; Howlader et al. [19] detected vertical collusion in bidding by constructing an SNA network model of individuals, organizations, communities and other participants and achieved good results; Van Den Heuvel [20] deterred bidding stakeholders' willingness to collude by feature analysis of vertical collusion in bidding and trace to the master and follower of bidding combined with genetic algorithm. Scholars also considered the psychology of participants [21] and the probability density function of auction price [22], etc. on collusion prevention.

To sum up, most of the studies on collusion in bidding of construction projects are focused on the analysis of collusion subjects and influencing factors, while the studies on evaluating and determining collusion tendency are relatively rare. In view of the constant change of vertical collusion in bidding for construction projects, more difficulty in collusion detection, unavailability of the evaluating data, deficiency in sample, and complex correlation among indicators, a comprehensive evaluation model of the tendency of vertical collusion in bidding for construction projects was developed based on deep neural network (DNN). Firstly, through literature research, file summarization, case analysis, and expert consultation, 18 evaluation indicators were determined for the tendency of bidders, tenderers, and bid evaluation experts to collude; secondly, a comprehensive evaluation model based on deep neural network was developed, and 130 cases were collected as the training set and test set of DNN model input data; at last, the stable DNN model could effectively evaluate the tendency of vertical collusion in bidding, which can help to prevent vertical collusion targetedly.

## 2. Methodology

### 2.1. Data Collection

1. Literature review: In China National Knowledge Infrastructure (CNKI) and Web of Science (WOS), the keywords “collusion”, “bidding collusion”, and “bidding corruption” were searched. In order to avoid potential influence from age-old literature, 847 papers in the past 5 years (from 2015 to 2020) were chosen as data samples, including 291 from the general journal, 187 from master or doctor thesis, and 369 from the core and above journals.
2. Summarization of court files: In the study of bid collusion, court files give sufficient resources of real cases, so it is necessary to make full use of this data source. For its case abundance and authenticity, bid conspiracy registered in China Judgements Online from 2015 to 2020 were researched and summarized in this paper.  Table 1 shows some cases of crimes.
3. Typical case analysis: The typical cases of bidding were searched and summarized from the Chinese government procurement network, Chongqing public resources trading network, and other websites.  Table 2 shows some typical examples of collusion on the website.

### 2.2. Expert Consultation

By qualitatively analyzing and summarizing the collected collusive data, five experts in the field of bidding in China were consulted on the vertical collusion among the tenderers, bidders, and bid evaluation experts.  Table 3 shows the profile of the expert panel. Three specific questions were included. Generalized indicators were extracted by recording and analyzing the original expert responses.

  Question 1: What do you think are the general manifestations or behaviors of tenderers when they are involved in collusion?
  Question 2: Based on the bidders' behavior provided by us, what do you think will the bidders do when they are involved in collusion?
  Question 3: In your opinion, what are the main bias practices of bid evaluation experts in bidding activities?

### 2.3. Deep Neural Network

The main shallow machine learning models are Support Vector Machines (SVM) [23], boosting models [24], and maximum entropy models [25], etc. The emergence of BP algorithms has effectively promoted the development of deep neural network represented by Multi-Layer Perceptron (MLP) [26]. Compared with shallow machine learning models, deep neural network models are characterized by deep network layers, large number of network model parameters, and strong learning ability, which has triggered a wave of scholars' research in this field. For example, Zhu and Shan [27] established a high-dimensional neural network model to comprehensively evaluate the probability of public engineering project investment risk. Langkvist et al. [28] pointed out that the deep neural network has three advantages: breaking through data limitations, considering complex interactions, and avoiding overfitting problems. Takeuchi and Lee and Ding et al. [29, 30] both used deep neural network to explore the trend of stock price fluctuations, and verified the model through empirical research. Dixon et al. [31] have proven through a large number of cases that deep neural network has the advantages of fusion and analysis of multiple information, thus forming a more effective information set for follow-up research. Pei et al. [32] applied the white box testing framework to the deep neural network system to further improve the performance of the deep learning system. Ma et al. [33] transplanted the mature combined testing technology from traditional software testing to the deep neural network system, during the test, the technology of using combined test coverage to guide the generation of test cases was proposed and achieved good results. Sun et al. [34] proposed a set of relatively complete and systematic test standards based on the characteristics and applicability of deep neural network, which provided strong support for follow-up research, etc. DNN is a neural network model with several hidden layers added, also known as MLP. Among several common structures of deep learning, DNN is superior in strong feature extraction ability, simple model structure, low training difficulty, and fast convergence speed, etc. Considering the problems that the data of the indicators for comprehensive evaluation of vertical collusion in bidding of construction projects are not easy to obtain, insufficient sample size and complex interrelationship, as well as the characteristics and requirements of comprehensive evaluation of tendency of vertical collusion, this study used DNN model to conduct the comprehensive evaluation.

#### 2.3.1. Structure of DNN

Deep neural network generally consists of an input layer, a number of hidden layers, and an output layer (as shown in Figure 1), and the layers are fully connected to each other, i.e., any neuron in layer *i* must be connected to any neuron in layer *i* + 1. In terms of the small local model, the data in DNN, same as perceptron's, is transferred among different neurons by linear function *z*=∑*w*_*i*_*x*_*i*_+*b* and function *σ* (*z*), where xi represents the input from the *i*th neuron, *w*_*i*_ is the connection weight of the *i*th neuron, and *b* represents the offset, and the learning process of the neural network is essential to continuously adjust the connection weights and neuron offsets between the neurons to get closer to the output of the training samples.

#### 2.3.2. Application of DNN

The training and testing process of deep neural network includes training, determining parameters, testing, and checking network accuracy (as in Figure 2).

### 2.4. Research Flow

Specific to small data set, this paper developed the model by employing DNN method and transfer learning algorithm, in which the obtained tendency evaluation value of tenderers, bidders, and bid evaluation experts were as input. Transfer learning can apply the knowledge learned in a domain or a task to another domain or task. Given a source domain Ds and a learning task Ts in the source domain, a target domain Dt and the corresponding learning task Tt, the goal of transfer learning is to use the knowledge in Ds and Ts to complete the task Tt in Dt. This method can be used when there is insufficient data. Combining the transfer learning with deep neural network can reduce the sample size requirement of DNN model, so as to adapt to the small dataset of vertical collusion in bidding in order to obtain a high comprehensive evaluation accuracy. The flow of the developed evaluation model is shown in Figure 3.

## 3. Results

Based on the keywords in literature, collusion in typical cases, and the causes in the court files, the frequency of collusion of bidders and tenderers is plotted as shown in Figure 4.

Based on the collected keywords of collusive practices of bidders and tenderers, the three questions were interviewed to experts and their original judgment was recorded. Grounded on the collated expert consultation results, indicators and explanations were reached for evaluating actors in construction projects bids, shown in Table 4. The range of model input values for all indicators was [1, 10].

## 4. Development of the DNN Model

### 4.1. Data input

In this study, a total of 130 cases were collected (due to the large number of participants, only the data of the top 5 bidders were obtained for each case), and divided into two parts: training samples and testing samples. In terms of the ratio of training and test sample settings, Zhang and Zhao [35] set 90% as the training set and 10% as the test set when building a neural network model of user Q&A-related variables and monthly sales of clothing; Wen et al. [36] randomly divided the data into 80% of the training set and 20% of the test set when building a neural network with effective wave height inversion set; Ding et al. [37] used the improved lion swarm algorithm to optimize the neural network model for the housing price prediction problem by using the first 70% of the data samples as training samples and the last 30% as test samples, etc. In view of the concealment of vertical collusion in bidding, the correlation among monitoring indicators and the difficulty in obtaining indicator data, this study took about 60% training samples and about 40% test samples, i.e., 75 training samples (former 60 collusive cases and latter 15 non-collusive cases) and 55 test samples (former 40 collusive cases and rest 15 normal cases) (see Table 5).

### 4.2. Transfer Learning

A parameter-based transfer learning approach was used in this study, on the premise that some parameters or prior distributions were shared between the source and target tasks model. The algorithm achieved knowledge transfer by finding these shared parameters or prior distributions and processing them. The unique advantages of transfer learning have caused widespread application by scholars: Liao et al. and Liu et al. [38, 39] used the transfer learning algorithm to complete the text detection task and the edge detection task on the basis of the visual geometric group network structure; Wu et al. [40] used the transfer learning algorithm to control the ship name identification, and considerable test results were obtained. Considering the concealment of vertical collusion in bidding and the complex relationship between indicators, the study improved the model with the help of parameter transfer algorithm, aiming to improve the accuracy of vertical collusion evaluation.

In the tendency evaluation analysis, Hu [41] studied electricity consumption characteristics and constructed a tracking monitoring model for electricity theft users with the help of improved BP neural network to conduct deep monitoring of electricity users. The main reasons for using this model as a transfer learning source were: (1) the similarity of electricity consumption characteristics and vertical collusion evaluation indicators as source domains; (2) the outputs of the two models are basically the same, one is the theft suspicion coefficient, and the other is the tendency of vertical collusion; (3) the indicator data is readily available from inner system of an electric power company, where the electricity consumption data is abundant and easily accessible; hereafter, the specific process of the comprehensive evaluation model based on transfer learning algorithm in this study, see Figure 5.

Among them, the fine-tuning method of the model was as follows: the relevant parameters of the source model were transferred to the target model; the weights of some layers were fixed to adjust the weights of other layers, and the process was repeated until the error between the output value of the model and the actual value meets the requirements; at this time, the optimal weights between layers were obtained. Suppose there were P samples to train, where *X*_*pi*_ = the *i*th input value of *p*, *n*, *q*, *m* = the respective number of nodes in each layer, *V*_*ki*_ = the weight from node *i* in the input layer to node *k* in the hidden layer, *w*_*jk*_ = the weight from node *k* in the hidden layer to node *j* in the output layer, and the activation function was the sigmoid function. The forward input process of this model network is as follows.

The output from input layer to the hidden layer is

(1) $$\begin{array}{c} Z_{pk}=g\left({\text{net}}_{pk}\right),\\ =g\left(\sum_{i=0}^{n}v_{ki}-x_{ki}+\theta_{k}\right),\;k=0,1,2,\ldots ,q. \end{array}$$

The output from the hidden layer to the output layer is

(2) $$\begin{array}{c} Y_{pk}=g\left({\text{net}}_{pj}\right),\\ =g\left(\sum_{k=0}^{q}w_{jk}z_{pk}+\theta_{j}\right),\;k=0,1,2,\ldots ,m. \end{array}$$

The total model error is

(3) $$\begin{array}{c} E=\sum_{p=1}^{P}E_{p},\\ =\frac{1}{2}\sum_{p=1}^{P}\sum_{j=1}^{m}{\left(t_{pj}-y_{pj}\right)}^{2}. \end{array}$$

where *E*_*p*_ = the sample error, *t*_*pj*_ = the expected output, and *y*_*pj*_ = the model output.

The inverse process uses the gradient descent method to adjust the weight values, and the calculation process is as follows.

The weights between layers are updated as follows:

(4) $$\begin{array}{c} \Delta w_{jk}=-\eta \frac{\partial E}{\partial w_{jk}},\\ =\eta \sum_{p=1}^{P}\left(-\frac{\partial E_{p}}{\partial w_{jk}}\right),\\ =\eta \sum_{p=1}^{P}\left(-\frac{\partial E_{p}}{\partial {\text{net}}_{pj}}•\frac{\partial {\text{net}}_{pj}}{\partial w_{jk}}\right). \end{array}$$

where *η* = the learning rate.

The output layer error is

(5) $$\begin{array}{c} \delta_{pj}=-\frac{\partial E_{p}}{\partial {\text{net}}_{pj}},\\ =-\frac{\partial E_{p}}{\partial y_{pj}}•\frac{\partial E_{pj}}{\partial {\text{net}}_{pj}}. \end{array}$$

The hidden layer node weights are updated as:

(6) $$\begin{array}{c} \Delta v_{ki}=-\eta \frac{\partial E}{\partial v_{ki}},\\ =\eta \sum_{p=1}^{P}\left(-\frac{\partial E}{\partial v_{ki}}\right),\\ =\eta \sum_{p=1}^{P}\left(-\frac{\partial E_{p}}{\partial {\text{net}}_{pk}}•\frac{\partial {\text{net}}_{pk}}{\partial w_{ki}}\right). \end{array}$$

The hidden layer error is

(7) $$\begin{array}{c} \delta =-\frac{\partial E_{p}}{\partial {\text{net}}_{pk}},\\ =-\frac{\partial E_{p}}{\partial z_{pk}}•\frac{\partial z_{pk}}{\partial z_{pk}}. \end{array}$$

### 4.3. Training and Testing of Network

#### 4.3.1. Transfer of the Benchmark Network Structure

In this study, the configuration 10-6-1(number of inputs-number of hidden layer neurons-number of output) of DNN model for tracking and monitoring electricity theft users was used as the benchmark network structure based on the transfer learning algorithm to develop a DNN model for comprehensive evaluation [41], and the benchmark network parameters are shown in Table 6.

#### 4.3.2. Optimization and Training

For the characteristics of the evaluation of bidding vertical collusion tendency, the transferred benchmark network was debugged in this study, specifically: considering the small sample size of the evaluation indicators of the participants in the vertical collusion and the data correlation is more complicated, increased network dimensions, and adjusted the number of neurons. The compact network structure is conducive to get the optimal conclusion through less training data. Due to the difference in collusion evaluation indicators among bidders, tenderers, and bid evaluation experts, two different network structures were designed to match the comprehensive evaluation; the configuration of tenderer & bidder network. The training parameters of DNN-based comprehensive evaluation model for bidders, tenderers, and bid evaluation experts are finally determined in Table 7.

Specifically, the mean squared error MSE was generally chosen as loss function for the training of DNN models, as shown in the following equation.

(8) $$\begin{array}{c} \text{MSE}=\frac{1}{mp}\sum_{r=1}^{p}\sum_{j=1}^{m}\left({\hat{y}}_{rj}\right.{\left.-y_{rj}\right)}^{2}, \end{array}$$

where *m* = the number of output nodes, ${\hat{y}}_{rj}$  = the expected output value of the network, *p* = the number of training samples, and *y*_*rj*_ = the actual output of the network. Sigmoid, the activation function of hidden layer and output layer, also functioned as threshold function of neural network, mapped its variables to interval from 0 to 1 with input interval whole real number and output internal [0, 1], satisfying the designed need for comprehensive vertical collusive evaluation. The expression of the sigmoid function is shown in the following equation.

(9) $$\begin{array}{c} f\left(x\right)=\frac{1}{1+e^{-x}}. \end{array}$$

According to the training results, the configuration of the developed model is obtained as shown in Figure 6.

In this study, the Python 3.9 code was implemented for model training, and the output target value of collusion case was set as any value in [0.3, 1] and the output target value of normal case was set as any value in [0, 0.3] during training [42].

In the tenderer and bidder network structure, the input layer was the value of the vertical collusion indicator of tenderer and bidder, value range [1, 10], input randomly based on actual situation; the hidden layer, the optimal number determined by constant adjustment, was 2 layers with 4 and 2 neurons, respectively; the output layer was any value in tenderer and bidder collusion tendency interval (0, 1). In addition, in movement of twice dimension reduction in achievement of higher accuracy for tendency evaluation, the weight distribution matrices were matrix 8 × 4 and 4 × 2, respectively. In the 3rd dimension degradation, the weight distribution matrix from *L*3 to *L*4 was matrix 2 × 1 with [0.169, −0.317] in tender network and matrix 2 × 1 with [0.404, 0.827] in bidder network.

Since there were only 4 indicators for evaluating the collusion behavior of bid evaluation experts, this paper adjusted the dimensions of the comprehensive evaluation DNN network towards experts referring to the DNN network for tenderers and bidders. In the bid evaluation expert network structure, the input layer was the value of the bid evaluation expert vertical collusion indicators, value range [1, 10], input randomly based on actual situation; the hidden layer, the optimal number determined by constant adjustment, was 1 layer with 2 neurons; the output layer was any value in bid expert collusion tendency interval (0, 1). In reach of high accuracy for comprehensive tendency evaluation model in bid evaluation expert's party, the weight distribution matrix in first dimension reduction was matrix 4 × 2, the second dimension, namely, from *L*2 to *L*3, was matrix 2 × 1 with [0.044, 0.075].

#### 4.3.3. Gradient Descent of the Error

Since the loss function used in the model was the minimized loss function, the model output error could be solved by gradient descent algorithm. In this study, the number of iterations was set to 2000 when training the developed model, and it was found that the mean square error of training samples was close to 0 (see Figure 7). Thus, the final determined network parameters and weight distribution matrix could reflect that the developed model was regarded as reliable. In this study, in order to alleviate or avoid the problem of overtraining, an early termination algorithm was carried to mitigate overfitting, i.e., the training was terminated as soon as the overfitting trend of the model was detected.

#### 4.3.4. Testing

The test was conducted using the aforementioned 55 test samples, and the results are shown in Table 8. The experimental results showed that the developed model predicted 48 correct and 7 incorrect, with a comprehensive accuracy of 87.3%, which was high, further indicating that the model could be regarded as reliable and accurate.

## 5. Model Application and Discussion

### 5.1. Background

In bid evaluation of a provincial highway mainline site construction project, the expert panel finally locked 4 candidates, in the order of *A*1, *A*2, *A*3, and *A*4. The project department determined the first and the second winning candidates according to the number of labor teams to be recruited and the recommended order of winning candidates.

Combined with the obtained evaluating indicators of the tenderers, bidders, and bid evaluation experts, the following improper practices were found in the bidding activity after repeated review and continuous retroactive tracking of the indicators by the government supervisory department: (1) in the process of preparing bidding documents, the tenderers added “special technology”, and “enterprise qualification”, and the scoring criteria and scoring indicators in bid evaluation part were unreasonable; (2) in the bidding process of *A*1, the tenderer leaked relevant bidding information to the enterprise before bidding announcement, what was more, the tenderer used his position to inform the enterprise of important information about the required materials; (3) during the bidding process of *A*2, the tenderer set “limited number system” pre-qualification conditions for him; selected the bid evaluation experts at his will, and finally designated his next bid evaluation experts by the enterprise; (4) *A*3 and *A*4 participated in the bidding in accordance with normal procedures, and no abnormalities were found in the indicators; (5) during bid evaluation, the bid evaluation team deliberately gave *A*2 high score at tenderer's instruction, and made obvious tendentious remarks.

### 5.2. Comprehensive Evaluation of the Tendency of Vertical Collusion

Wu [42] established a model for measuring the strength of the tendency of bidders and tenderers to collude based on evidence-based reasoning approach, and concluded that the strength level could be divided into weaker (0–0.3), weak (0.3–0.5), strong (0.5–0.8), and stronger (0.8 – 1), and the strong level reflect the existence of collusion between the two parties. Through comparative analysis, in this case, the collusion evaluation level is as shown in Table 9, which provides some theoretical reference significance for the comprehensive evaluating level of the tendency of collusion of the model output value.

The input values of the model are shown in Table 10, each caught by three regulatory experts' investigating and tracking indicators of the tenderer, 4 bidders, and bid evaluation experts.

The above three sets of values were applied to the developed model and run in Python 3.9, respectively, and the results are shown in Table 11.

Based on the output results, we could get that there was a high probability of collusion in the bidding activity, and the colluding subjects were the tenderers, *A*1 bidder, *A*2 bidder, and bid evaluation experts.

### 5.3. Discussion

Based on the tendency indicators of vertical collusion in bidding and the comprehensive tendency model of vertical collusion, four types of prevention suggestions for vertical collusion in bidding can be put forward, namely, routine prevention, early warning prevention, moderate prevention, and severe prevention.

1. Routine prevention faces the situation that the actors are labeled weaker with the developed model. Preventive measures are mainly routine check, irregular check, special check, and emphasized check to materials and practices of the body of tenderer, bidder, and bid evaluation expert in the implementation process.
2. Early warning prevention suits for monitoring the weak assessed by the developed model, and the preventive measures are mainly to monitor the whole process of bidding activities dynamically, compare bidding data at multiple levels, and review bidding problems in all aspects with the help of intelligent technologies such as 5 G communication network, Internet of Things, and cloud computing. At the same time, the blockchain multi-point storage technology for data confidentiality management, identification system to strengthen expert management and other intelligent technologies can combine to guarantee the whole process, multi-level and all-around strict review of bids, judges, evaluation, and management of bidding activities in construction projects.
3. Moderate prevention applies to those scored strong doers evaluated by the developed model, and the preventive measures mainly include the implementation of commitment system, joint and several penalty system and heavy fine system. In addition, giving full play to the advantages of trading platform facilities and resources and real-time interaction of network information, it is suggested that the relevant supervisory department and government legal department should reasonably reorganize the business process to effectively prevent collusion in construction bidding.
4. Severe prevention adapts to the stronger participants marked by the developed model, and the preventive measures mainly include introducing social credit code system and weaving a detailed and sound credit record system for those bidding-related parties. With this system, any relevant activities are always observed, recorded, and exposed on the designated platform haunting psychology of daring not collusion. Moreover, expending supervision role of public service and third party, constantly innovating supervisory ideas, improving supervisory methods, and maintaining supervisory concepts, all are organically bonded to a systematic supervision mechanism to monitor the whole stage of bidding.

## 6. Conclusions

This study developed a deep neural network model for comprehensive evaluation of the tendency of vertical collusion with the help of transfer learning, subdivided to 4-layer model (8-4-2-1) for tenders, 4-layer model (8-4-2-1) for bidders, and 3-layer model (4-2-1) for bid evaluation experts. The collected 130 cases were trained and tested to the established DNN model, and the result of 87.3% accuracy said the model was reliable. Depending on comprehensive evaluation results of the model, four types of collusion prevention suggestions are proposed: routine, early warning, moderate, and severe. The specific measures for routine prevention include routine check, irregular check, special check, and emphasized check; early warning prevention include strengthening the audit strength of participating parties, improving the transparency of bidding activities, and popularizing intelligent technology; the moderate prevention are mainly implementing the commitment system, strengthening the public reporting channels, and improving electronic bidding; the severe prevention falls on temporary inclusion in blacklist, encouraging joint departmental supervision, and establishing a new regulatory mechanism bridging the whole bidding process. The comprehensive evaluation model of tendency of vertical collusion behavior developed in this study has some reference value for the standardization of bidding market in China and other countries.

Since the comprehensive evaluation executed in this study needs to fully consider various factors, the study needs to be further explored and improved, mainly in the following two aspects: on one hand, the differences in corporate culture and local customs have not been taken into account when obtaining the comprehensive evaluation indicators, which need to be considered in future research; on the other hand, there is some subjectivity in data collection by using expert consultation as input value, thus subsequent collection means of evaluation data waits for deep exploration to be close to actual situation.

## Figures and Tables

**Figure 1:** DNN basic structure.

**Figure 2:** DNN basic implementation process.

**Figure 3:** Research flow.

**Figure 4:** Indicator frequency of tenderers and bidders' collusion.

**Figure 5:** Parameter transfer process.

**Figure 6:** Configuration of the developed model.

**Figure 7:** Training effect.

**Table 1:** Cases of bid conspiracy crimes in China judgements online (partial).

No.	Release date	Case	Case no.	Court name
1	July.7 2020	Tenderers used the convenience of their jobs to illegally accept property from bidders for their benefit.	(2020) No.2 Yue crime	Guangdong high People's court
2	Oct.2 2020	Bidders borrowed the qualifications of other enterprises to obtain qualifications.	(2020) No.53 11*E* crime	Huanggang intermediate people's court, Hubei province
3	Aug.31 2020	Bidders borrowed qualifications, agreed on bid prices, and participated in bidding.	(2020) No.67 05 Zhe crime	Zhejiang Huzhou intermediate people's court
4	June.28 2019	Tenderers and bidders negotiated on bid prices, programs, and other contents before bidding	(2019) No.2181 supreme court civil	Supreme people's court of the people's republic of China
5	Nov.6 2019	Bidders bribed tenderers in return for bid information before bid publicity.	(2019) No.1507 01 Yue crime	Guangzhou intermediate people's court, Guangdong province
6	Dec.31 2019	Being a member and leader of the bid evaluation committee, the bidder participated in whole process of the evaluation.	(2019) No.5242 supreme court civil	Supreme People's court of the people's republic of China
7	Sep.21 2018	Bid evaluation experts made use of their job convenience to make profit for bidders for illegal properties against bid evaluation regulation.	(2018) No.7 0921 chuan crime	Pengxi county people's court
8	Dec.6 2018	Bidders undertook projects in the form of bidding after obtaining information about bidding in advance from the tenderers.	(2018) No.1055 0103 Hei crime	Harbin Nangang district people's court

**Table 2:** Bidding collusion cases (partial).

No.	Publishing platform	Collusive practice	Company name
1	https://www.ccgp.gov.cn/	Provide false materials to win bid	XX Co., Ltd.
2	https://ggzyjyjgj.cq.gov.cn/	Bid evaluation experts were inclined to the intended bidders.	XX Co., Ltd.
3	https://www.ccgp.gov.cn/	Bidders provided false materials to meet the tender requirements.	XX Greening Co., Ltd.
4	https://jycg.hubei.gov.cn/	Tenderers used their positions or power to unintentionally or intentionally authorize bid evaluation experts to give high scores to specific bidders.	XX environmental construction Co., Ltd.
5	Other sites	Tenderers broke the rules to facilitate intended bidders	XX consulting Co.

**Table 3:** Profile of the expert panel.

Employer	Position	Years of experience	Largest project ever managed/consulted
Contractor	Project manager	19	RMB ¥ 1.1 billion
Consultant	Deputy manager	16	RMB ¥ 3.5 billion
Academia	Professor	20	RMB ¥ 64 million

**Table 4:** Comprehensive evaluation indicator system.

Subjects	Indicators	Indicator description
Tenderer	Valid bid ratio *X*_11_	The ratio of valid bids to total bids. The range of value is 0–100%. The tenderer, on purpose of boosting cooperative bidder's success rate, may reduce the valid bid rate in some way to let the activity less competitive.
	Selection of tendering method *X*_12_	Dismemberment (unreasonable) or normal bidding activities (reasonable). One is to split project to evade due tender procedure, and the other is to set specific conditions to change the public tender to invited tender, awarding “benefits” to collusive bidders.
	Tenderers convey tendentious information *X*_13_	Yes or no. The tenderers pass project-related information to collusive bidders or persuade other bid evaluation experts privately to make the related enterprise win the bid.
	Release timeliness of bidding information *X*_14_	Some tenderers may change the tender release time for collusive bidders' consideration, resulting in information not accessible simultaneously to advance winning rate.
	Setting reasonability of technical parameter *X*_15_	Some unreasonable arrangements, for instance, changing range value to specific value, may be done towards to bidders by tenderers.
	Tendency of tender requirements *X*_16_	Tenderers may require previous business contacts such as construction performance or similar project experience as tender premise to preclude other participants.
	Extra credit bias *X*_17_	Tenderers may set unreasonable qualification conditions such as the size of registered capital, geography, years of operation, and employees in bid preparation as a way to increase the evaluation score of collusive bidders.
	Rationality of evaluation setting *X*_18_	Normally evaluation in bid documents should be made in regard to actual project situation, past experience, and relevant regulations, practically the tenderers may set inclined standard and unscientific weight to favor collusive bidders.

Bidder	Bid winning rate *X*_21_	The residual difference indicator is examined. When the residual difference between the actual and predicted winning bids falls outside a certain interval, it indicates that the bidder has a tendency to collude with the tenderers partly.
	Special requirements compliance *X*_22_	The conformity of unreasonable conditions such as the scale of registered capital, geographical area, years of operation, and employees in tender.
	Reassessment rate *X*_23_	The value range is 0–100%. When the supervisory authority finds that the bidder's conditions are consistent with the evaluation factors listed in the agreements or that the bidder has unreasonable practices, it will ask the experts to re-evaluate.
	Authenticity of bidding materials *X*_24_	Yes or no. During the review of the bidders' materials, the tenderers may know the materials have problems but keep silent, and then tacit collusion of both sides occurs.
	Similarity of technical bid parameters *X*_25_	The value range is 0–100%. The technical content similarity between tender party and bidder party, expressed as the overlapping content accounting for the total technical content.
	Fitness to business documents *X*_26_	The value range is 0–100%. The degree of business conformity (such as project performance, and enterprise qualification) specified in tender documents, expressed as similar content accounting for total content of the business bid.
	Type of bidder risk appetite *X*_27_	Aggressive, positive, balanced, robust, and conservative. Risk appetite has a significant positive effect on the tendency of collusion, and aggressive risk appetite further stimulates the occurrence of collusive practices.
	Degree of mastery of key project information *X*_28_	The tenderers may deliberately conceal key information about the project and only let collusive bidders know the information to ensure their dominance in the bid evaluation process.

Bid evaluation expert	Deviation of expert score *X*_31_	The deviation range is examined. There are horizontal deviation and vertical deviation. The experts may be suspicious of collusion when two deviations exceed the range (±10% ∼ ±20%).
	Reward strength of bid evaluation *X*_32_	The strength of rewards for bid evaluation experts largely reflects whether experts adopt collusive practice, and the greater the strength of rewards based on previous good evaluations, the less likelihood experts' collusion will occur.
	Rigor of bid evaluation process *X*_33_	In the bid evaluation process, the experts select the team leader randomly; the experts are guided by the tenderer's comments and actions and do not question the bid evaluation methods or the experts make targeted remarks.
	Expert type *X*_34_	Randomly selective experts are tested on personality and psychological scales, and then define according to results as 4 types: Capricious, ambitious without knowledge, independent, and opinion leader, with sequence of decrease in collusion.

**Table 5:** Data set classification.

Sample type	Quantity (abnormal & normal)
Training sample	75 (60 + 15)
Test sample	55 (40 + 15)
Total	130

**Table 6:** Training parameters of the Benchmark network.

Parameter	Value
Configuration	[10, 6, 1]
Number of layer (*n*)	3
Activation function of hidden layer	Sigmoid
Learning rate	0.02
Loss function	Mean squared error (MSE)
Iteration	2000
Output layer activation function	Sigmoid

**Table 7:** Training parameters of the developed DNN model.

Parameter	Value	
Configuration	Tenderer&Bidder	[8, 4, 2, 1]
	Expert	[4, 2, 1]
Number of layer (*n*)	Tenderer&Bidder	4
	Expert	3
Activation function of hidden layer	Sigmoid	
Learning rate	0.5	
Loss function	MSE	
Iteration	2000	
Output layer activation function	Sigmoid	

**Table 8:** Accuracy of model test results.

Case collusion type	Total	Incorrect number	Correct rate (%)
Tenderer & bidder & expert	11	2	81.82
Tenderer & bidder	21	2	90.48
Bidder & expert	8	0	100
Normal	15	3	80

**Table 9:** Collusion evaluation level.

Participate	Evaluation levels and collusion tendency intervals			
Tenderer	Stronger [0.84, 1]	Strong [0.39, 0.84)	Weak [0.23, 0.39)	Weaker [0, 0.23)
Bidder	Stronger [0.76, 1]	Strong [0.30, 0.76)	Weak [0.23, 0.30)	Weaker [0, 0.23)
Expert	Stronger [0.85, 1]	Strong [0.50, 0.85)	Weak [0.25, 0.50)	Weaker [0, 0.25)

**Table 10:** Inputs for the model (3 regulatory experts).

Indicator	*X*_11_	*X*_12_	*X*_13_	*X*_14_	*X*_15_	*X*_16_	*X*_17_	*X*_18_
Tenderer	5, 5, 5	3, 4, 3	7, 7, 8	4, 5, 5	8, 7, 8	8, 7, 7	6, 5, 6	8, 8, 7

Indicator	*X*_21_	*X*_22_	*X*_23_	*X*_24_	*X*_25_	*X*_26_	*X*_27_	*X*_28_
Bidder *A*1	3, 3, 4	8, 7, 7	1, 1, 1	1, 2, 2	9, 9, 9	8, 8, 8	6, 6, 6	6, 5, 5
Bidder *A*2	3, 3, 3	8, 7, 8	1, 1, 1	2, 1, 1	8, 8, 8	7, 7, 7	5, 5, 5	6, 5, 6
Bidder *A*3	3, 3, 3	6, 5, 4	1, 1, 1	1, 2, 1	5, 5, 5	4, 4, 4	4, 4, 4	6, 6, 5
Bidder A4	2, 2, 2	6, 5, 5	1, 1, 1	1, 1, 1	4, 4, 4	4, 4, 4	4, 4, 4	4, 3, 3

Indicator	*X*_31_		*X*_32_		*X*_33_		*X*_34_	
Expert	7, 8, 7		4, 3, 5		8, 7, 8		6, 6, 7	

**Table 11:** Output values of the model (3 regulatory experts).

Output	Tenderer	Bidder *A*1	Bidder *A*2	Bidder *A*3	Bidder *A*4	Bid evaluation expert
Expert 1	0.8559	0.8083	0.7053	0.2019	0.2456	0.7997
Expert 2	0.8553	0.8089	0.7055	0.2023	0.2458	0.8001
Expert 3	0.8562	0.8091	0.7049	0.2020	0.2451	0.7998

## Data Availability

The data used to support the findings of this study are available from the corresponding author upon request.
